The article "An Artificial Neural Network-Based Approach to Optimizing Energy Efficiency in Residential Buildings in Hot Summer and Cold Winter Regions" was retracted in 2023. Reasons: unreliable results or conclusions; concerns about the data; concerns about the results or conclusions; concerns about the peer review.

# An Artificial Neural Network-Based Approach to Optimizing Energy Efficiency in Residential Buildings in Hot Summer and Cold Winter Regions

**DOI:** 10.1155/2022/2611695

**Published:** 2022-08-25

**Authors:** Mingyue Gao

**Affiliations:** School of Art and Design, Shaanxi Fashion Engineering University, Xi'an, Shaanxi 712046, China

## Abstract

Resource depletion and ecological crisis have prompted human beings to reflect on the behavior patterns based on industrial civilization so as to seek ways of sustainable development of human society, economy, technology, and environment. The energy consumed in the construction process, commonly known as building energy consumption, accounts for more and more of the total social energy consumption, and with the continuous development of social economy and the improvement of living standards, this proportion will be larger and larger. The structure of the neural network directly determines its performance and work efficiency. The structure optimization of the neural network is not only a hot issue in this field but also an insurmountable key step in engineering applications. With the increase of network depth, the structural optimization difficulty index of the neural network increases, so solving this problem has important theoretical and practical significance for the design and application of the neural network. In this paper, the energy saving of buildings is optimized based on the optimization of structures such as particle swarm optimization (PSO) algorithm and restricted Boltzmann machine. The experimental results show that the BPNN optimized by the improved PSO algorithm is significantly better than the non-optimized BPNN and the BPNN optimized by the basic PSO algorithm. The comprehensive output rate of the optimized neural network can reach 64.5%. In general, the error rate of the optimized artificial neural network (ANN) will be 57.65% lower than the original one.

## 1. Introduction

As one of the three high energy-consuming industries, which keep pace with industry and transportation, in the global energy consumption [1]. From the perspective of building energy consumption composition, the energy consumption of public buildings is mainly concentrated in air conditioning system, elevator, and other auxiliary equipment [2]. Urban residential energy consumption is mainly composed of cooking, household appliances, air conditioning, lighting, and domestic hot water. Construction activity is one of the largest activities of human transformation of nature [3]. The progress of industrial technology has realized the absolute control of the architectural space environment, which has led people to make full use of energy and various natural resources and constantly meet the increasing demand for the quality of the artificial environment [4]. However, tracing back to the source of the energy crisis and environmental deterioration, it is found that the energy resources consumed by human construction activities and the pollutants emitted account for 30% of the total social volume [5]. However, because the previous architectural design failed to fully consider building energy conservation, it had to mainly rely on heating and equipment to improve the indoor thermal comfort environment, and it also required a lot of energy consumption [6]. According to the actual situation of hot summer and cold winter areas, this paper calculates the energy saving of solar power generation, biomass energy, lighting, solar hot water, and solar floor heating. Considering economic and social benefits and other factors, the electrical energy-saving evaluation model is established and trained by ANN. The network has good generalization performance and high accuracy of evaluation, which provides a scientific basis for the implementation of energy-saving transformation [7]. In areas with hot summer and cold winter, the summer is extremely hot, the winter is humid and cold, and the air humidity is high. Building energy conservation is the key to energy conservation and emission reduction in my country. However, building energy conservation should not be at the expense of the comfort of living. Considering the health and comfort of the living environment, building energy conservation is efficient and meaningful [8]. In this paper, people's feelings about the climate environment are divided into three situations: first, comfortable, then acceptable, and finally unacceptable [9]. Building energy conservation is a systematic project, and all factors influence and restrict each other. Because the evaluation model results of the existing building energy efficiency index system are too abstract, the usability of the evaluation information contained in it is low, and it cannot play its due role in building energy efficiency evaluation. An “acceptable” climate environment refers to a climate environment that is acceptable from both physical and psychological aspects without significantly affecting people's work efficiency and quality of life, including people's adaptive behaviors such as appropriately increasing or decreasing clothes and normal physical reactions such as a small amount of sweating [10]. In hot summer and cold winter areas, the indoor and outdoor temperature difference in winter is generally only half of that in cold areas, and the influence of the shape coefficient on winter energy consumption is half less than that in cold areas. In addition, residents in this area often have to open windows for ventilation in winter and hope to strive for more passive means such as natural ventilation to dissipate heat in summer. Therefore, it is easy to form such a view, that is, as one of the important indicators of building energy conservation. Although there are differences in the climate and environment that different people can accept, this difference is obviously much smaller than the climate and environment that different people can tolerate [11]. Because a BP model can be described by a finite number of parameters, it can be expressed by a finite length string code. After transforming the parameter code of BP into the string of genetic algorithm, an appropriate performance evaluation function can be selected, and then GA can be used for global search in the parameter space. This method can achieve a better balance between regional exploration and spatial expansion. At the beginning of genetic search, the crossover operation of random population tends to expand the search space in a wide range. With the acquisition of high fitness solutions, the crossover operation tends to explore around these solutions.

The ANN model is the basis of deep learning, and in engineering applications, the hyper parameters of the ANN structure directly affect the ability of the model to solve problems, and directly determine the actual working effect of the trained model in the industry [12].

Based on this, this paper mainly studies the application of ANN in residential building energy-saving optimization in hot summer and cold winter areas, in order to give full play to the effect of ANN technology in residential building energy-saving optimization methods and the development of residential building energy-saving optimization methods. The main purpose of this paper is to optimize the structure of artificial PSO.

## 2. Methodology

### 2.1. Research Based on ANN

BP neural network (BPNN) belongs to the feedforward neural network [13]. BPNN is the most widely used neural network at present. Its algorithm and model are relatively mature. The prediction results predicted by BPNN have reliability and credibility [14]. The structure of BPNN is simple, and the learning and training algorithms are relatively mature. For multi-layer BPNN, appropriate weights and activation functions can be used to approximate any nonlinear mapping to any degree. The general structure of the neural network is shown in Figure 1.

The shape factor refers to the ratio of the outer surface area to the volume required to contact the atmosphere in the enclosed room of the building [15]. The thermal performance of the building envelope is mainly analyzed from the three aspects of roof, exterior wall, and window, and the interior walls of doors and stairs are approximated as exterior walls. For roofs and exterior walls, two indexes, heat transfer coefficient and thermal inertia, are used, of which the average heat transfer coefficient is used, that is, the heat transfer coefficient of the exterior wall is obtained by the area-weighted method; the heat transfer coefficient and shading coefficient indexes are used for windows. The window-to-wall area ratio is the ratio of the area of the window opening to the area of the exterior wall of the room facade unit. Since the heat inside the building is dissipated through the envelope structure, the heat transfer is related to the heat transfer area of the outer surface. The smaller the shape coefficient, the less the way of heat dissipation, and the more the energy-saving significance. For a single hidden BPNN, its internal forward calculation is as follows:

(1) $$\begin{array}{c} t_{m}=\sum_{m}\omega_{mi}O_{i}+\theta_{m},\\ O_{m}=f\left(t_{m}\right)=\frac{1}{1+\exp\left(-t_{m}\right)}. \end{array}$$

The output of the input layer node *i* is equal to the input. In the above formula, *ω*_*mi*_ is the connection weight between the node *m* of the hidden layer and the node *i* of the input layer. *θ*_*m*_ is the bias or threshold of the hidden layer node *m*, and *f* is the Sigmoid function. The input and output of the output layer node *l* are

(2) $$\begin{array}{c} t_{l}=\sum_{m}\omega_{lm}O_{m}+\theta_{l}.\\ O_{l}=f\left(t_{l}\right)=\frac{1}{1+\exp\left(-t_{l}\right)}. \end{array}$$

In the previous formula, *ω*_*ml*_ is the connection right between the output layer node *l* and the hidden layer node *m*, and *θ*_*l*_ is the offset of the output layer node *l*.

The BP algorithm is obtained according to the principle of steepest descent, and the convergence speed is very slow. In practical applications, a momentum term is often added to improve the learning speed. The back-propagation process of the error is as follows:

The expression of the weight *ω*_*lm*_ between the output layer and the hidden layer is

(3) $$\begin{array}{c} \omega_{lm}\left(k+1\right)=\omega_{lm}\left(k\right)+\alpha \delta_{l}O_{m}+\beta \left[\omega_{lm}\left(k\right)-\omega_{lm}\left(k-1\right)\right], \end{array}$$

including *δ*_*l*_=*f*(*t*_*l*_)(*t*_*l*_ − *O*_*l*_). For the weight *ω*_*ml*_ between the hidden layer and the input layer, the expression is

(4) $$\begin{array}{c} \omega_{ml}\left(k+1\right)=\omega_{ml}\left(k\right)+\alpha \delta_{m}O_{l}+\beta \left[\omega_{ml}\left(k\right)-\omega_{ml}\left(k-1\right)\right]. \end{array}$$

Among them, *δ*_*m*_=*f*(*t*_*m*_)∑_*l*_*δ*_*l*_*ω*_*lm*_ is the number of iterations of *k*, *α* is the learning rate, that is, the gain coefficient of the weight, and *β* is the momentum coefficient, which is used to adjust the convergence rate.

The basic component of the neural network model is the neuron model, which allows multiple data to be input and a single datum to be output, and its way of processing input data is nonlinear [16]. The core goal of deep learning is to learn the input data through the model so that the deep neural network can show the specific feedback to the data, which can also be understood as that the model can make correct judgment on the target problem. The error of the network model fitting to the dataset is called the empirical error, and the judgment error of the samples outside the training dataset is called the generalization error, and minimizing the generalization error is the ultimate goal of model training. These characteristics together determine the working principle of the neural network model, and the connection and arrangement of neurons together constitute the main structure of the modern neural network model [17]. The neuron model with *i* input data is shown in Figure 2.

BPNN is a fully connected feedforward neural network, which is a network structure formed by combining neuron models in layers. The model uses the error of each forward calculation as the basis for parameter updating in the training process. The optimization method and the neural network model can make the loss function converge quickly during training, and express the target characteristics faster. BPNN and constrained Boltzmann machine structure optimization algorithm design. As the two important models of ANN, feedforward neural network and restricted Boltzmann machine provide an important training mechanism and optimization method for the rapid development of deep learning. For these two models, we study the structure optimization method of a fully connected network using information entropy and mean square error to describe the local and global working state of the network and adjusting the network structure according to the working state to make the model structure tend to be stable.

The restricted Boltzmann machine model is an important part of the deep belief network. Through its optimization of the model parameters in the pretraining process of the deep belief network, the feature extraction ability of the model and the input data and the parameter convergence speed are increased [18]. Most importantly, this enables the depth confidence network to complete the training task at almost any depth [19]. The restricted Boltzmann machine is a directed acyclic graph composed of two network layers, all of which are connected. The specific structure is shown in Figure 3.

When the input data is binary data, the model is Bernoulli restricted Boltzmann machine; when the input data is decimal, the model is a Gauss–Bernoulli restricted Boltzmann machine [20]. The neurons in the hidden layer are also binary and are obtained by Gibbs sampling after forward calculation.

Suppose there is a group of particles in the solution space, each particle has its own position and velocity, and the particles can exchange information [21]. When a particle searches for its own optimal solution, it can share the information of the optimal solution with the group. The group obtains a group optimal solution, and other particles move closer to the optimal particle according to the group optimal solution, continue to find a new optimal solution, and finally get a best result [22]. This is also the basic principle of the particle swarm algorithm. In the final analysis, the learning of ANN is the process of adjusting the parameters of the network itself. The main method is to continuously adjust its own system parameters by calculating the error according to the input and output data given by the outside world and directly calculate its own system parameters according to the specific requirements of the outside world.

Assuming that there are *n* particles in the *m*-dimensional search space, each particle has no weight and volume and flies at a certain speed in the search space, and the flying speed and direction can be dynamically adjusted according to the flying experience of individuals and groups.

For minimization problems, the smaller the objective function value, the better the corresponding fitness value.

Let the optimal position experienced by all particles in the particle swarm be *P*_*g*_(*t*), which is called the optimal position of the swarm. Then,

(5) $$\begin{array}{c} P_{g}\left(t\right)\in \left\{P_{0}\left(t\right),...,P_{s}\left(t\right)\right\}|f\left(P_{g}\left(t\right)\right)=\min\left\{f\left(P_{0}\left(t\right)\right),\ldots ,f\left(P_{s}\left(t\right)\right)\right\}. \end{array}$$

The basic particle swarm algorithm evolution formula is

(6) $$\begin{array}{c} v_{ij}\left(t+1\right)=v_{ij}\left(t\right)+c_{1}r_{1j}\left(t\right)\left[P_{ij}\left(t\right)-x_{ij}\left(t\right)\right]+c_{2}r_{2j}\left(t\right)\left[P_{gj}\left(t\right)-x_{ij}\left(t\right)\right]\\ x_{ij}\left(t+1\right)=x_{ij}\left(t\right)+v_{ij}\left(t+1\right). \end{array}$$

Here, *v*_*ij*_(*t*) represents the speed of the *i*th dimension and the *j*th iteration of the *t*th particle, and *x*_*ij*_(*t*) represents the position of the *i*th dimension and the *j*th iteration of the *t*th particle; *P*_*ij*_(*t*) represents the individual optimal position of the *i*th particle at the *j*th iteration, and *P*_*gj*_(*t*) represents the group optimal position of the *j*-th iteration of the *t*th dimension of all particles in the particle swarm; *c*_1_,  *c*_2_ represent two acceleration constants; two random numbers are generated in the *r*_1*j*_(*t*),  *r*_2*j*_(*t*) iteration of *j* dimension representing all particles of *t* particle swarm; and *r*_1*j*_(*t*) ∈ [0,1],  *r*_2*j*_(*t*) ∈ [0,1] are independent of each other.

### 2.2. Structural Characteristics and Climatic Conditions of Residential Buildings in Areas with Hot Summer and Cold Winter

From the perspective of outdoor climate, in the whole country, areas with hot summer and cold winter are not the worst environment, winter is far less cold than severe cold areas, and summer temperature is slightly lower than that of hot summer and warm winter areas [23]. For this reason, for a long time in the past, hot summer and cold winter areas were defined as non-heating areas, and there were almost no heating and air-conditioning residential buildings in this area. As a result, the indoor environmental quality in this area is the worst in China [24]. In summer, although the windows are open, the wind is often very small or even non-existent. The indoor temperature during the day is almost the same as the outdoor temperature, and the indoor temperature drops very slowly at night, and the air humidity is high, which is abnormally sultry, often making people sleepless at night. In winter, due to the low sunshine rate, the indoor humidity is high [25]. In order to avoid the breeding of bacteria, the windows must be opened for ventilation from time to time, so the indoor and outdoor temperatures are almost the same. It is not uncommon to get sick or frostbitten by cold. Tables 1 and 2 are the statistics of the proportion of two- and three-bedroom residential buildings in a residential area in hot summer and cold winter.

Through a large number of human experiments, the relationship equations between the above six parameters and the prediction of human thermal sensation under the condition of steady-state thermal environment are proposed, and the prediction average thermal sensation voting model is a classical model in the field of human thermal comfort research. However, the calculation of PMV is extremely complex, so the parameters are not easy to measure. Although the pMv index represents the feeling of the vast majority of people in the same environment, due to the existence of climate differences and individual differences, the pMV index cannot represent the feeling of people in China, and it is not suitable for human thermal comfort models in areas with hot summers and cold winters.  Table 3 is the thermal sensory scale for PMV values.

Thermal comfort research is to solve the thermal comfort index by using multiple influencing factors. Therefore, RBFNN is selected as the method to establish the human thermal comfort model in hot summer and cold winter areas. The network establishment process is as follows:

The input vector is *X*=[*x*_1_, *x*_2_,…,*x*_6_]^*T*^, the hidden layer vector is *R*=[*r*_1_, *r*_2_,…, *r*_6_], and the expression is

(7) $$\begin{array}{c} R_{j}=\exp\left[-\frac{{\left\|X-C_{j}\right\|}^{2}}{2\sigma_{j}^{2}}\right]. \end{array}$$

The *K*-means clustering algorithm is used to determine the center vector *C*_*j*_ and the base width vector *σ*_*j*_, and the supervised learning algorithm is used to obtain the weight vector *W*_*j*_ of the network. Then, the mathematical expression of the output of the network, that is, the thermal comfort model, is as follows:

(8) $$\begin{array}{c} f\left(x\right)=\sum \exp\left[-\frac{{\left\|X-C_{j}\right\|}^{2}}{2\sigma_{j}^{2}}\right]\times W_{j}. \end{array}$$

The ability of the PSO algorithm to optimize the neural network can generally be judged according to the performance of the trained neural network. BPNN is generally used to classify specific objects or perform function fitting, so there are four main indicators for optimizing BPNN for PSO:

Let the total number of training samples to be classified be *M*, and a total of *m* samples show classification errors during the training of BPNN; then the classification error rate of training samples is

(9) $$\begin{array}{c} \varepsilon_{Train}=\frac{m}{M}\times 100\%. \end{array}$$

Assuming that the total number of test samples to be classified is *N*, and the BPNN has a total of *n* samples with classification errors during training, the classification error rate of the training samples is

(10) $$\begin{array}{c} \varepsilon_{Test}=\frac{n}{N}\times 100\%. \end{array}$$

The mean square error of the training sample is

(11) $$\begin{array}{c} MSE_{Train}=\frac{1}{M}\sum_{i=1}^{M}{\left(Y-Y^{\prime }\right)}^{2}. \end{array}$$

The mean square error of the test sample is

(12) $$\begin{array}{c} MSE_{Test}=\frac{1}{N}\sum_{i=1}^{N}{\left(Y-Y^{\prime }\right)}^{2}. \end{array}$$

When using BPNN to solve the classification problem, the performance indexes of these four test neural networks can be used. When using BPNN for function approximation and function fitting, the first two performance indicators cannot be used, and only two performance indicators, TrainMSE and TestMSE, can be used.

## 3. Result Analysis and Discussion

In order to obtain scientific, reasonable, and accurate conclusions, this paper will express the frequently encountered nonlinear model with BPNN. This paper operates by setting the nonlinear unknown model as a black box. First, the BPNN is trained with the input and output data of the system so that the BPNN can fit the unknown system, and then the trained BPNN can be used to predict the output of the system. Therefore, this paper also needs to set parameters, which will be set as learning rate *η*=0.2 and learning goal *ε*=0.00002. The PSO algorithm is introduced for comparison.  Figure 4 and Figure 5show the analysis diagrams of non-optimized BPNN and optimized BPNN on training sets A and B, respectively.

According to the above analysis, it is obvious that the optimized BPNN has better output effect in the analysis of the non-optimized BPNN and the optimized BPNN. On the unoptimized BPNN, we can find that the fluctuation of the graph is relatively large, which will have a greater impact on the experimental analysis and specific operations. Although there are parts higher than 50%, it is still lower than 50%. The output efficiency of the optimized BPNN is above 40% on the whole, which will also ensure a good effect in actual operation. The comprehensive output rate of the optimized neural network can reach 64.5%.

Based on the above experimental analysis, this paper will continue the experiment. The ANN error rate before and after optimization and the neural network error based on the PSO algorithm are analyzed (experimental sets *s* and m), as shown in Figures 6 and 7.

In the optimization process of BPNN, the PSO algorithm is integrated, and the convergence speed and robustness of particles are obviously improved in the evolution process. However, the convergence of particles is lower than that of the original PSO. For the non-optimized BPNN, the average value of the square sum of errors of the test samples is 4.514, and the variance is 1.524. The data distribution is relatively concentrated. For the BPNN optimized by the PSO algorithm, the average value of the sum of squares of the error of the test samples is 3.254, which is significantly lower than that without optimization; the variance is 7.584; and the data distribution is relatively scattered. The BPNN optimized by the PSO-HS algorithm has the smallest mean value of the sum of squares of errors, which is 1.547, and the variance is 0.4512. The data are all between 2 and 3, and the distribution is the most concentrated. Generally, the error rate of the optimized ANN will be reduced by 57.65% compared with the original one.

## 4. Conclusions

With the rapid development of economy, the continuous increase of building area, the rapid growth of household appliances, and the increase of energy consumption of heating and air conditioning have caused the continuous increase of building energy consumption, and building energy conservation has become an increasingly urgent issue. Green building is an important means to realize sustainable development, save resources and energy, and protect the environment. This paper discusses the problems that the ANN is easy to fall into the local optimal solution, optimizes the connection weight of BPNN by the genetic algorithm, and obtains a more accurate and practical BPNN for the prediction of residential building energy consumption and indoor comfort. The basic method of the neural network for energy-saving evaluation is as follows: Through feature extraction, select the parameters that are more sensitive to building energy-saving as the input vector of the network, and the energy-saving evaluation index as the output, establish the energy-saving classification training sample set, and then train the network. The PSO algorithm is applied to the optimization of BPNN weights, and the optimized BPNN is fitted with a nonlinear function. The experimental results show that the BPNN optimized by the improved PSO algorithm is significantly better than the non-optimized BPNN and the BPNN optimized by the basic PSO algorithm. The comprehensive output rate of the optimized neural network can reach 64.5%. In general, the error rate of the optimized ANN will be 57.65% lower than the original one.

## Figures and Tables

**Figure 1:** Structure diagram of a general neural network.

**Figure 2:** Neuron model.

**Figure 3:** Restricted Boltzmann machine.

**Figure 4:** Analysis of unoptimized BPNN.

**Figure 5:** Optimized BPNN analysis.

**Figure 6:** Analysis of the ANN error rate before and after optimization.

**Figure 7:** Neural network error analysis based on particle swarm algorithm.

**Table 1:** Statistical table of the length-width ratio of two types of households.

Breadth length ratio	0.3	0.5	0.7
Building number	1	14	24
Percentage	1.7	25.7%	36.1%

**Table 2:** The ratio of three types of households and the statistical table of buildings.

Specific value	0.4	0.6	0.7
Building number	1	14	15
Percentage	3.4	36.4	52.1

**Table 3:** Thermal sensation scale of the PMV value.

PMV value	−2	−1	0	1	2
Hot feeling	Cool	A little cold	Suitable	A little hot	Warm

## Data Availability

The data used to support the findings of this study are available from the author upon request.
